The article "University Archives Autonomous Management Control System under the Internet of Things and Deep Learning Professional Certification" was published in 2022. Journal: Comput Intell Neurosci.

# University Archives Autonomous Management Control System under the Internet of Things and Deep Learning Professional Certification

**DOI:** 10.1155/2022/4854213

**Published:** 2022-09-21

**Authors:** Yue Ma, Bing Dai, Baorong Ding

**Affiliations:** The School of Civil Engineering, Harbin University, Harbin 150086, China

## Abstract

The current work aims to meet the needs of the development of archives work in colleges and universities and the modernization of management to realize the standards and standardization of all aspects of archives business construction in colleges and universities, so as to improve the political and professional quality of archives cadres. First, the radio frequency identification (RFID) technology based on the Internet of things (IoT) digitizes the university archive labels. Meanwhile, the filing cabinet's intelligent security system preserves confidential files. Second, the convolutional neural network (CNN) algorithm under deep learning is introduced and college profile information is identified. Finally, the concept of professional certification is used to clarify the purpose of the university archives automation management system. Different activation functions are used to analyze the recognition accuracy loss and recognition accuracy of university archives. The identification error of You Only Look Once (YOLO) of the ReLU-convolutional neural network (R–CNN) of college archives is analyzed. The results show that the selection of rectified linear units (ReLU) activation function for CNN can effectively reduce the loss of identification accuracy of college archives and can improve the accuracy of identification of college archives. The algorithm based on the ReLU activation function has a smaller recognition error accuracy in college archives than that of the YOLO algorithm. The recognition error of the YOLO algorithm is slightly higher than that of the R–CNN. The font recognition error of archival information based on the R–CNN is relatively large. However, the conclusion is reasonable due to the recognition difficulties of handwritten archival fonts. The file positioning recognition error rate is 19.00%, the file printing font recognition error rate is 4.75%, and the image recognition error rate is 1.90%. These results have a certain reference value for the process of identifying information in the automatic management of university archives by CNN under different activation functions.

## 1. Introduction

At present, there are many problems in the management of university archives. Many grassroot units have not formulated and implemented detailed rules for filing archives and lacked standardized operating procedures. The objectives of normative management of archives are not clear, the arrangement of archives lacks unified classification and enforceable standards, and the processing of archives is unscientific. These circumstances have resulted in a low degree of standardization in the generation, collection, filing, archiving, classification, grouping, and in numbering and cataloging of archives. The archived materials are not uniform, and it is difficult to fully reflect the school's teaching management level and teaching quality [1–3]. Most of the staff have not undergone professional archival knowledge training and do not understand the importance of archives, the requirements of archives management, the collection, arrangement, filing, and binding of archives materials, and their awareness of archives collection is weak. Moreover, most of the archives management personnel have several jobs and they do not devote enough energy to the archive's work. Some archived materials are not true and accurate enough, and the archived materials cannot be supplemented in a timely and accurate manner, so the archived materials cannot truly reflect the actual situation of the individual, resulting in incomplete file management [4–6]. Some schools overemphasize the construction of scientific research, the proportion of scientific research funds is large, and they do not pay attention to the archives' work, and the funds for the archives cause are insufficient. Some colleges and universities have not included the archives work funds in the planning ranks, and even if they are included in the planning, the proportion is very small [7, 8]. In view of the abovementioned problems in the archives management work, how to do a good job in the archives management of colleges and universities is an urgent problem that needs to be solved at present [9, 10].

The original meaning of the Internet of Things (IoT) refers to connecting all items to the Internet through information sensing devices such as radio frequency identification (RFID) to achieve intelligent identification and management [11]. The Computer Systems Laboratory of Binghamton University has carried out a variety of work on wireless sensors in mobile self-organizing network protocols, application layer design of sensor network systems, etc. [12]. Using the sensor network hardware node, UbiCell integrates sensors, microprocessors, wireless transceivers, and other embedded chips and has various functions such as information acquisition, signal processing, data transmission, and real-time monitoring. Its wireless multimedia sensor network node has an image acquisition and processing capability of 300,000 pixels and 60 frames per second (FPS), which is sufficient to meet the application requirements of network monitoring and identification [13]. Researchers started a RFID-related electromagnetic theoretical research. The publication of those researches led many commercial companies to develop application equipment suitable for electronic artide surveillance (EAS) but it can only be used to identify targets. For detection, no more tags can be stored, so when there are multiple object tags present, the monitoring system cannot identify the identified item [14–16]. The United States initially applied RFID technology to the transmission industry and access control, while Europe used short-range monitoring RFID technology for animal monitoring [17]. The concept of “deep learning” first entered people's field of vision because of its powerful feature extraction capabilities and flexibility. The LeNet network architecture forms the current form of the convolutional neural network (CNN) and has achieved excellent results on the Mixed National Institute of Standards Technology (MNIST) handwritten digit recognition dataset [18].

In order to efficiently identify the information of university archives automatically and to reduce the waste of human resources, the current work digitizes college archives tags from IoT-based RFID technology. Meanwhile, it provides an intelligent security system for filing cabinets to preserve confidential archives. Second, it introduces the CNN algorithm under deep learning and provides information on college archives. Moreover, the purpose of the university archives automation management system is clarified through the concept of professional certification. Finally, for different activation functions, the university archives are analyzed for the loss of recognition accuracy and the accuracy of recognition. You Only Look Once (YOLO) of the ReLU-convolutional neural network (R–CNN) is used for error analysis of college file recognition. The current work has a certain reference value for the process of identifying information in the automatic management of university archives by CNN under different activation functions. The innovation is that the file identification is different from the traditional identification method, and the identification accuracy of college files under different activation functions is tested, which reduces the difficulty of identifying files. The combination of the rectified linear units (ReLU) activation function with the CNN structure can effectively identify different characters in the file and can identify consecutive characters.

Section 1 is the introduction, which illustrates the existing problems of archives management in colleges and universities and provides the research background. Then, this part also explains the research status of the IoT and deep learning technology, and finally, the research method process is described.  Section 2 is the theoretical part, which explains the importance of the professional accreditation concept in the archives management of colleges and universities.  Section 3 is the research method part, which expounds on the application of RFID technology, CNN, and contract lock in the archives management system of colleges and universities, respectively.  Section 4 is the result part, which shows the recognition accuracy loss and recognition accuracy of different activation functions for college archives, as well as the analysis of the identification error of college archives by R–CNN YOLO.  Section 5 is the discussion, which discusses the research results and illustrates the feasibility.  Section 6 is the conclusion, describing the research results and expounding on the research shortcomings and future development directions.

## 2. The Concept of Professional Certification of University Archives

There are strict confidentiality management regulations for all kinds of students, teaching, personnel, and scientific research files in colleges and universities. In order to prevent the occurrence of modern signatures and leakage of information in the archiving process, contract locks are used to authenticate the real identity of the filers and ensure their signatures. Additionally, the concept of professional accreditation is used to strengthen the management control of the university archives system. The concept of professional certification is shown in Table 1.

## 3. Methods

### 3.1. The IoT-The Application of RFID in the Archives Management System of Colleges and Universities

IoT refers to various devices and technologies through various information sensing devices, such as sensors, RFID technology, a global positioning system (GPS), infrared sensors, laser scanners, and gas sensors. These devices and technologies can collect any object or process that needs to be monitored, connected, and interacted within real-time, and collects all kinds of information such as sound, light, heat, electricity, mechanics, chemistry, biology, and location and combines them with the Internet to form a huge Internet. Its purpose is to realize the connection between things and things, things and people, and all things and the network, which is convenient for identification, management, and control. RFID technology can support fast reading and writing, nonvisual identification, mobile identification, multitarget identification, positioning, and long-term tracking management [19]. RFID is not limited by size and shape in reading and does not need to match the fixed size and printing quality of paper for reading accuracy. RFID tags have the characteristics of miniaturization and various forms, making them applicable to different products.

RFID technology is an important part of the IoT perception layer. It is a technology that uses RF-radio frequency signals to realize contactless information transmission through spatial electromagnetic coupling and achieves object recognition through the transmitted information. Common RFID products are inductive electronic chips, inductive cards, contactless cards, electronic labels, and electronic barcodes. A complete RFID system consists of a reader and a transponder. Its action principle is that the reader transmits infinite radio wave energy of a specific frequency to the transponder, which is used to drive the transponder circuit to send out the internal ID code. The reader at this time will receive this ID Code. The principle of RFID identification is shown in Figure 1.

In Figure 1, RFID is mainly composed of an electronic label, an antenna, and a reader. There are two data areas in the electronic tag chip, namely, the identification (ID) area and the user data area. The ID area is used to store the globally unique identification code, the user identifier (UID). USD is stored in read only memory (ROM) when making chips and cannot be modified. The user data area is for users to store data, which can be read, written, and modified or added operations. Meanwhile, the antenna is a device that realizes the spatial propagation of RF-radio frequency signals and establishes a wireless communication connection. The language of communication between RFID and the reader is electromagnetic waves. Each time the reader sends a signal of a certain frequency through the antenna, after receiving the signal, the identification information stored in the electronic tag is transmitted through the wire, and the reader will receive it through the antenna. Moreover, we identify the information sent back by the electronic tag, and finally, the reader will send the identification result to the host, so that the purpose of identification is achieved. The RFID-based university archives management system is shown in Figure 2.

In Figure 2, the initialization of the RFID electronic label is completed by the RFID printer. The electronic label is gradually bound to all the data information in the electronic archives of the university as a unique identifier for the query archives. RFID readers are installed on the channels entering and exiting the archives management center of the university. When the files enter and leave the general file management center of the university, the reader will identify the file information by reading the electronic tag data and complete the rapid acquisition of the file entry and exit data. When the archives are transferred to other departments, the information of the incoming archives can be accurately proofread through the configured mobile collection equipment, and the inflow of the archives can be completed quickly and accurately. The intelligent filing cabinet manages some confidential files and realizes the functions of authorized pickup, real-time inventory, and remote monitoring. Based on this, the smart filing cabinet is processed with preventive measures. The intelligent security system of the intelligent filing cabinet is shown in Figure 3.

In Figure 3, each smart filing cabinet has an independent electronic lock control and an unauthorized personnel cannot open the filing cabinet. The whole cabinet is equipped with a video surveillance device and the school can design an alarm strategy. The school can link the security system to carry out alarm settings for mobile phone alarms, network alarms, and other alarm methods, to ensure the security of college confidential files in all-round way and improve the file prevention rate.

### 3.2. Positioning and Information Identification of University Archives Based on Deep Learning

Deep learning refers to a collection of algorithms that use various machine learning algorithms to solve various problems such as images and texts on multilayer neural networks. The core of deep learning is feature learning, which aims to obtain hierarchical feature information through hierarchical networks, to solve the important problems that required the manual design of features in the past. Deep learning is a framework that includes a variety of algorithms. Among them, the CNN is a kind of neural network specifically designed to process data with a grid-like structure. Convolutional networks are those neural networks that use convolution operations instead of normal matrix multiplication operations in at least one layer of the network. The CNN is essentially a filter. The filter is filtered by convolution. CNN work well with other types of models, such as recurrent neural networks and autoencoders, one example of which is symbolic language recognition. To some extent, the CNN tries to regularize on the basis of a feed-forward neural network (FNN) to prevent overfitting, and it can also identify the spatial relationship between data well [20]. The network structure of a simple CNN is shown in Figure 4.

In Figure 4, the CNN employs a convolutional function. The neurons between layers are not used for the connection. The convolutional layer connects the neurons in the part between the four layers. It consists of convolutional layers, pooling layers, and fully connected layers. Among them, the convolution layer cooperates with the pooling layer to form multiple convolutional groups, extract features layer by layer, and finally complete the classification through several fully connected layers. To sum up, CNN simulates feature distinction through convolution and reduces the order of magnitude of network parameters through weight sharing and pooling of convolution. Finally, traditional neural networks are used for tasks such as classification [21]. First, the image data of the archive page size A4 paper are input based on the archive image. The archive data label is shown in the following equation:

(1) $$\begin{array}{c} y={\left[P_{c},b_{x},b_{y},b_{w},b_{h},c_{1},c_{2},c_{3}\right]}^{T}\text{.} \end{array}$$

In equation (1), *P*_*c*_ is 1 and there is a target (picture, file printing font, and file information font). *b*_*x*_, *b*_*y*_, *b*_*w*_, and *b*_*h*_ are the horizontal and vertical coordinates of the center position of the image frame. The length and width of the border, *c*_1_, *c*_2_, and *c*_3_ are the target categories. The loss function is as follows:

(2) $$\begin{array}{c} y=\left[1,b_{x},b_{y},b_{w},b_{h},1,0,0\right]\text{.} \end{array}$$

Convolution implements sliding window and realizes image window traversal. We constructed a subset of images to be recognized based on archive images and constructed a joint training set. The relationship between the size of the output layer and the size of the input layer, filter size, and step size is shown in the following equation:

(3) $$\begin{array}{c} output=\left[\frac{input-filter+1}{stride}\right]\text{.} \end{array}$$

In equation (3), *output* is the size of the output layer. *Input* is the size of the input layer. *Filter* is the size of the filter. *Stride* is the step size. The joint training set includes a subset of archival images to be identified and a subset of archival images. The computation of convolutional image features is shown in equations (4) and (5):

(4) $$\begin{array}{c} f=Re\text{LU}\left(\overset{10}{\underset{i=1}{\sum }}x_{i}w_{i}\right)\text{,} \end{array}$$

(5) $$\begin{array}{c} ReLU=f\left(x\right)=\left\{\begin{array}{cc} \alpha x\text{,} & x<0,\\ x\text{,} & x\geq 0\text{.} \end{array}\right. \end{array}$$

When the convolutional image features are calculated, let the sliding window stride=1. Re*LU* is a symbolic function. *x*_*i*_ is the file image feature data. *w*_*i*_ is the connection weight. *f* is the output value. *α* is a parameter. In addition, the activation function can also choose *sigmoid* and *tanh*, as shown in the equations (6) and (7):

(6) $$\begin{array}{c} f\left(x\right)=\frac{1}{1+e^{-x}}\text{,} \end{array}$$

(7) $$\begin{array}{c} \begin{array}{cc} \tanh\left(x\right)=\frac{\sinh\;\left(x\right)}{\cosh\left(x\right)\;} & =\frac{x^{x}-x^{-x}}{e^{x}+e^{-x}} \end{array}\text{.} \end{array}$$

The height and width of the archive image output are shown in equations (8) and (9):

(8) $$\begin{array}{c} h=\frac{I\_h-c\_h}{stride\_h}+1\text{,} \end{array}$$

(9) $$\begin{array}{c} w=\frac{I\_w-c\_w}{stride\_w}+1\text{.} \end{array}$$

The input file image size is *I*_*w∗I*_*h*=210*∗*297. The sliding window step size is stride_*w* and stride_*h*. *c*_*w∗c*_*h* is the size of the convolution kernel. Multiple convolution kernels produce multiple convolutional feature maps. The output feature size is as follows:

(10) $$\begin{array}{c} M=\frac{I_{w}*I_{h}-F+2P}{stride}+1\text{.} \end{array}$$

*M* is the feature size of the output file image. *F* is the size of the convolution kernel. *P* is the pixel filled in the feature map. According to the variance of the target image, the picture area of the image to be identified, the file text printing area, and the student information text area to which the file belongs are distinguished. At this time, the classification category is *k* = 3. SoftMax is used to classify and identify different file information, and its function expression is as follows: as

(11) $$\begin{array}{c} P\left(y=c|x\right)=\frac{1}{1+\sum_{k=1}^{c-1}e^{\theta_{k}^{T}x}}\text{.} \end{array}$$

In equation (11), *c*[*c* = 0, 1, 2] represents the type of classification. *X* is the variable value under different categories. *θ* is the surrogate estimated parameter. Intersection-over-Union, the concept used in IoU target detection is the overlap rate between the candidate bound and the ground truth bound, that is, the ratio of their intersection and union. The ideal situation is complete overlap, that is, a ratio of 1. Let *C* be the real frame of the file, *G* be the algorithm predicted frame, and its calculation is as follows:

(12) $$\begin{array}{c} LoU=\frac{area\left(C\right)\cap area\left(G\right)}{area\left(C\right)\cup area\left(G\right)}\text{.} \end{array}$$

### 3.3. Application of Contract Lock in the University Archives Automation Management Control System

Archives management is one of the important basic tasks of colleges and universities. According to the “Administrative Measures for Archives of Colleges and Universities,” colleges and universities shall file nearly ten kinds of archives materials such as students, teaching, personnel, administration, party and mass, scientific research, and equipment promptly every year. With the advancement of file management informatization, more and more colleges and universities have begun to introduce electronic signatures to promote the comprehensive digital transformation of file transfer and filing. The university archives automation management control system can be seen in Figure 5.

In Figure 5, the contract lock electronic signature system is open and integrated with the university archives management system and the school affairs management system to provide legal and effective electronic signature and electronic seal services for the transfer and filing of archives in the school [22]. Whether it is an electronic file or a paper file, the filing approval can be initiated through the process. The archivist signs and seals online, which comprehensively improves the efficiency of university file transfer and filing. When thousands of documents are signed in batches, covenant lock provides batch signing services. The archive files in the archiving stage are unified and aggregated. Archivers can add electronic signatures in batches with one click, and the system will automatically affix a special stamp for archiving. In this way, the filer can be freed from the mechanized signing work, and the intelligent conversion of document specifications can be realized. Colleges and universities have strict requirements on the specifications of archived files, and business personnel must adjust according to the requirements before they can approve the filing. To improve the efficiency of file specification conversion, contract locks can intelligently select the specification style and can automatically adjust it.

## 4. Results and Discussion

### 4.1. Loss and Accuracy Analysis of University Archives Recognition under Different Activation Functions

According to the aforementioned research methods, the identification of university archives is analyzed for identification loss and accuracy.  Figure 6 shows the analysis of the accuracy loss of university file recognition under different activation functions.

As can be seen in Figure 6, the tanh activation function profile recognition accuracy loss is smaller than that of the ReLU activation function and less than the Sigmoid activation function. The tanh activation function profile has the smallest loss of recognition accuracy, with an average value of 0.16. Followed by the ReLU activation function, with an average recognition accuracy loss of 0.19. The largest loss is seen in the Sigmoid function, and the average loss of recognition accuracy in college archives is 0.38, and with the growth of the archive dataset, the degree of loss is uneven. Therefore, the ReLU activation function is chosen.  Figure 7 shows the accuracy analysis of university archives recognition under different activation functions.

As shown in Figure 7, the growth of the archive dataset and the archive recognition rate under different activation functions do not have much effect. The recognition accuracy of the ReLU activation function is similar to that of the tanh function. The sigmoid function is not very accurate in identifying university archives. The average file recognition accuracy of the ReLU function is 0.95, the file recognition accuracy of the sigmoid function is 0.89, and the file recognition accuracy of the tanh function is 0.96. Therefore, the recognition accuracy of ReLU and tanh functions is the best.

### 4.2. R-CNN and YOLO's University File Recognition Error Analysis

YOLO can use a fully connected layer at the end to predict dossier bounding boxes. Among them, the height of the bounding box is relative to the size of A4 paper, and because there are objects of different sizes and aspect ratios in each file image, it is difficult for YOLO to learn to adapt to the shapes of different objects during training, which leads to poor performance of YOLO in precise localization. YOLO draws on the prior box of faster-CNN's region proposal network (RPN). The PRN is used to convolve the feature map obtained by the CNN feature extractor to predict the bounding box and confidence (whether or not there is an object) at each location. Each location is set with a priori boxes of different sizes and scales. All RPN predicts are the offset of the bounding box relative to the prior, and using the prior makes learning easier. One of the pooling layers is removed to make the detection box resolution higher. The size of the input in the detection model is 210 ∗ 297. The total step size for downsampling in the YOLO model is 32. Therefore, the feature map size is 7 ∗ 9, and there is only one central position. The center point of some large objects falls in the center of the image, and it is relatively easy to use a center point of the feature map to predict the bounding box of the object. According to the automatic management and control system of university archives, R-CNN and YOLO are subjected to different degrees of recognition accuracy error analysis in the five categories of file printing fonts, file pictures, simulation, location, and file information fonts.  Figure 8 shows the error analysis of R-CNN and YOLO's university file recognition.

As shown in Figure 8, the algorithm using the ReLU activation function has a smaller error in the recognition accuracy of university archives than that of the YOLO algorithm. The font recognition error of archive information under R-CNN is the largest, which is 71.60%. However, there are difficulties in recognition based on handwritten archival fonts, so it is reasonable. In the process of simulating file recognition, the recognition error rate of R-CNN is 6.75% smaller than that of YOLO. Moreover, in the file positioning and recognition, the recognition error rate of R-CNN is 19.00% and the recognition error rate of YOLO is 32.65%. The recognition error rate of R-CNN in archivally printed fonts is 4.75% and the error rate is small. The error rate of YOLO in the file printing font is 13.60%. In the image recognition analysis, the R-CNN recognition error rate is 1.90% and the YOLO recognition error rate is 4.00%.

## 5. Discussion

The CNN under the ReLU activation function can effectively identify the character information of college archives. Harinahalli Lokesh and BoreGowda used deep learning technology to locate and recognize handwritten archives and found that deep learning technology could recognize continuous meteorological texts with a recognition accuracy of over 99.70% [23]. The conclusion not only shows that the use of CNN can identify university archives information but also that the identification effect is relatively consistent. This study analyzes the identification accuracy errors of different degrees in five categories of college archives' printing fonts, archive pictures, simulation, location, and archive font information, which can better reflect the effective path of identification and management of college archives.

## 6. Conclusion

Based on the IoT and deep learning methods, the university archives automation management and control system is studied under the concept of professional certification. The results show that the selection of the ReLU activation function for CNN can effectively reduce the loss of identification accuracy of college archives and can improve the accuracy of identifying college archives. In the analysis of the identification error of different categories of university archives, the font identification error of the archive's information under R-CNN is the largest, which is 71.60%. However, there are difficulties in recognition based on handwritten archival fonts, so it is reasonable. In the file location recognition, the recognition error rate of R-CNN is 19.00%, and the recognition error rate of YOLO is 32.65%. The recognition error rate of R-CNN in archivally printed fonts is 4.75% and the error rate is small. The error rate of YOLO in the file printing font is 13.60%. In the image recognition analysis, the R-CNN recognition error rate is 1.90% and the YOLO recognition error rate is 4.00%.

This study has a certain reference value for the process of identifying information in the automatic management of university archives under different activation functions of CNN [24–26]. However, a large amount of data during the operation of the CNN will cause hardware dependencies such as the central processing unit (CPU), trying to improve the CNN algorithm for optimization. Additionally, in the process of identifying university archives, this study is carried out under the guarantee that the fonts are not polluted, and the altered fonts are not identified and located [27–33]. It is hoped that the accuracy of CNN in image and font recognition will be increased, so as to be accurately recognized in the archives management system of colleges and universities.

## Figures and Tables

**Figure 1:** Identification principle of RFID.

**Figure 2:** RFID-based university archives management system.

**Figure 3:** System for intelligent security of filing cabinets.

**Figure 4:** Structure of the CNN.

**Figure 5:** The control system for automatic management of university archives.

**Figure 6:** Analysis of the accuracy loss of college archives recognition under different activation functions.

**Figure 7:** Analysis of the accuracy of university file recognition under different activation functions.

**Figure 8:** Analysis of university archives recognition error analysis of R-CNN and YOLO.

**Table 1:** Philosophy of professional certification.

Basic idea	Stress mechanism
Student center philosophy	Taking students as the center, making resource allocation and teaching arrangements around the achievement of training objectives and graduation requirements of all students, and taking the satisfaction of students and employers as an important reference for a professional evaluation

Output-oriented philosophy	Emphasizes the learning outcomes achieved by students after professional teaching design and teaching implementation, and evaluates the effectiveness of professional education against the core competencies and requirements of graduates

Continuous improvement concept	Effective quality monitoring and continuous improvement mechanism, which can continuously track the improvement effect, and use it to promote the continuous improvement of the quality of professional personnel training

## Data Availability

The data supporting the current study are available from the corresponding author upon request.
